# Prognostic Significance of Serum Biochemistry Profile in Children With Severe Acute Malnutrition

**DOI:** 10.7759/cureus.31266

**Published:** 2022-11-08

**Authors:** Ganesh K Verma, Rajesh K Yadv, Ramesh Chand, Imran A Khan, Shashi Bhushan S Katiyar, Mukeshvir Singh

**Affiliations:** 1 Pediatrics, Uttar Pradesh University of Medical Sciences (UPUMS), Saifai, IND; 2 Pediatrics, Motilal Nehru (MLN) Medical College, Prayagraj, IND; 3 Community and Family Medicine, Baba Raghav Das Medical College, Gorakhpur, IND

**Keywords:** child mortality, serum biochemistry, marasmus, kwashiorkor, severe acute malnutrition (sam)

## Abstract

Background

Malnutrition is a condition caused by defective nutrition in which either deficiency or excess of energy, protein, or micronutrients cause any measurable adverse effects on tissues/body form (body shape, size, composition), function, and clinical outcome. Children with a weight-for-height below -3 standard deviations (SD) of the mean based on the WHO standards have a high risk of death exceeding nine-fold that of children with a weight-for-height above 1 SD. In severe acute malnutrition (SAM) liver function tests, renal function tests, and serum electrolytes are deranged but their correlation with the prognosis is not well defined. So, there was a need for a study to know the prognostic significance. For this purpose, the current study was conducted in the pediatric ward of Uttar Pradesh University of Medical Sciences (UPUMS), Saifai, UP, India.

Method

This is an observational cross-sectional study conducted in the Department of Pediatrics, UPUMS (Saifai, UP, India) from January 2018 to July 2019 after approval from the institutional ethical committee. We enrolled 100 children with SAM who fulfilled the inclusion criterion after obtaining proper and well-informed consent.

Result

We studied children aged six to 59 months. The mean age of admitted patients in our study was nearly 24 months (24.18 months). The median age that was most common at the time of admission is nearly 1 year (13 months). In our study relation of serum sodium and serum potassium with the survival of SAM was found statistically significant.

Conclusion

Severe acute malnutrition is both a medical and social disorder. The risk of mortality increases as the severity of malnutrition increases. High-risk cases can be identified and can be treated aggressively and on a priority basis. Serum electrolyte disturbances in SAM are one of the most important predictors of the severity.

## Introduction

Malnutrition refers to deficiencies, excesses, or imbalances in a person’s intake of energy and/or nutrients. Thus, malnutrition connotes both under-nutrition and over-nutrition [1]. Malnutrition is a condition caused by defective nutrition in which either deficiency or excess of energy, protein, or micronutrients cause any measurable adverse effects on tissues/body form (body shape, size, composition), function, and clinical outcome [2]. Protein-energy malnutrition (PEM) is a form of malnutrition that is defined as a range of pathological conditions arising from a coincident lack of dietary protein and/or energy (calories) in varying proportions, which may present as kwashiorkor or marasmus.

The World Health Organization (WHO) and United Nations Children’s Fund proposed diagnostic criteria for severe acute malnutrition (SAM) in children aged six to 60 months including any of the following: weight-for-height below -3 standard deviations (SD) or Z scores of the median WHO growth reference (2006); visible severe wasting; the presence of bipedal edema; mid-upper arm circumference (MUAC) below 115 mm. Children with a weight-for-height below 3 SD of the median based on the WHO standards have a high risk of death exceeding nine-fold that of children with a weight-for-height above 1 SD [3]. Similar studies using MUAC as diagnostic criteria showed that the risk of dying is increased below 115 mm [4]. In most developing countries, fatality rates from SAM remain between 20% to 30%, largely due to poor case management stemming from inadequate knowledge among health workers as well as the use of outdated protocols. Severe acute malnutrition presents with a common clinical triad of complications including hypoglycemia, hypothermia, and associated infections followed by electrolyte disturbances such as hypokalemia or hypomagnesemia and dehydration that requires proper assessment and timely correction for improving outcomes. The management of SAM depends on complications. Once the diagnosis is confirmed, careful assessment is done for complications such as severe edema, medical complications, lack of appetite, and danger signs as per the Integrated Management Neonatal and Childhood Illnesses (IMNCI) algorithm.

Severe acute malnutrition is both a medical and social disorder, and the medical problems of the child result in part from the social problems at home. Malnutrition is the result of chronic nutritional and emotional deprivation when, due to ignorance, poverty, or family problems, caregivers are unable to provide a child with adequate nutrition and care. Nearly two-thirds of undernourished children worldwide live in two regions: Sub-Saharan Africa and Southern Asia [5]. Therefore, with proper management of children with SAM, Millennium Development Goals 1 (to eradicate extreme poverty and hunger) and 4 (to reduce child mortality) can be effectively achieved [6]. In a developing country like India, proper management of children with SAM can have a significant impact on child mortality.

Malnutrition in children is widely prevalent in India and is an important predictor of child mortality. In India, the infant mortality rate has been reduced from 57/1000 live births to 41/1000 live births, and the under-five mortality rate from 75/1000 live births to 50/1000 live births as per National Family Health Survey-4 (NFHS-4, 2015-2016). Among nutritional parameters studies, under-weight and stunting have been reduced from 42.5% to 35.8% and 48% to 38.4%, respectively; however, wasting and severe wasting increased from 19.8% to 21% and 6.4% to 7.5%, respectively [7]. Despite our continuous efforts, the percentage increase in the incidence of SAM is alarming, as SAM itself has a direct and indirect influence on infant mortality and under-five mortality rates. Clinically severe forms of malnutrition like marasmus and kwashiorkor represent only the tip of the iceberg of the entire burden of malnutrition. In SAM, liver function tests, renal function tests, and serum electrolytes are deranged, although their correlation with the prognosis has not been well defined. Hence the need for a study to highlight the prognostic significance. For this purpose, the current study was conducted in the pediatric ward of Uttar Pradesh University of Medical Sciences (UPUMS), Saifai, UP, India.

## Materials and methods

Study population

This observational cross-sectional study was conducted in the Department of Pediatrics of UPUMS in western Uttar Pradesh from January 2018 to July 2019. The study was duly approved by the UPUMS Ethical Review Committee (approval no.: 791/UPUMS/Dean/2019-2020/E. C. No. 29/2018). Written and informed consent was taken from one of the parents or any other adult relative present. All patients with SAM (six to 59 months of age) admitted to the pediatric ward and who met the inclusion criteria were included in this study irrespective of their gender. 

Inclusion criteria

Children aged six to 59 months with SAM, who met any of the following criteria: weight-for-height less than -3SD, and/or visible severe wasting and/or, mid-upper arm circumference (MUAC) <11.5 cm and/or, nutritional edema on both feet.

Exclusion criteria

The following children were not included in the study: children having primary liver or kidney disease, i.e., chronic liver disease, chronic kidney disease, or other organic and metabolic disorders such as glycogen storage diseases, channelopathies, muscular dystrophies, diabetes mellitus, etc.; patient’s guardian not giving consent.

Sample size

Being an observational cross-sectional study, the formula used was n=4pq/e2 where n=sample size, p= positive character/prevalence of SAM, q= [1-p], e= allowable error.

The prevalence of SAM in India is 6.4%; the allowable error is taken to be 5%; therefore, our sample size turns out to be 95. We have taken a sample size of 100 patients.

## Results

We enrolled 100 children with SAM, aged six to 59 months in this study. Demographic details are compiled in Table 1. The mean age of admitted patients in our study was about 24 months (24.18 months). Fifty-one percent of patients were male while the remaining 49% were female, with most of the patients having rural residence (about 65%) because our institute is located in a predominantly rural area, and only 35% had urban (district level) or semi-urban (block level) residence. The median age i.e., the most common age at the time of admission, was around obe year (13 months). About 30% were fully immunized for age, 64% were not fully immunized for age, and 6% were unimmunized at the time of admission.

**Table 1:** Demographic profile of participants

Demographic profile		Number	Percentage
Age	Six to 12 months	42	42.0
	13 to 24 months	24	24.0
	25 to 59 months	34	34.0
Gender	Male	51	51.0
	Female	49	49.0
Residence	Rural	65	65.0
	Urban	35	35.0
Immunization status	Completely Immunized	30	30.0
	Partially Immunized	64	64.0
	Not Immunized/Unknown	6	6.0

Clinical characteristics are compiled in Table 2. Around 11% of participants presented with severe dehydration, 12 children were found to have bilateral nutritional edema, 60 had MUAC less than 11.5 cm, and 76 children had weight-for-height < -3 SD.

**Table 2:** Clinical features of participants MUAC: Mid-upper arm circumference

Clinical characteristics		Number	Percentage
Pallor	Absent	38	38.0
	Present	62	62.0
Icterus	Absent	95	95.0
	Present	5	5.0
Hydration	No Dehydration	67	67.0
	Some Dehydration	22	22.0
	Severe Dehydration	11	11.0
Edema	Absent	88	88.0
	Present	12	12.0
Weight-for-height	< -3 SD	76	76.0
	< 2 SD	24	24.0
	< 1 SD	0	0
MUAC (in cm)	<11.5cm	60	60.0
	>/= 11.5cm	40	40.0

In this study, 10% of the participants had hypoglycemia at the time of admission, total serum bilirubin was raised among 23%, albumin levels were low for age in 21%, while serum glutamic-oxaloacetic transaminase (S. SGOT) and serum glutamic pyruvic transaminase (S. SGPT) levels were raised in 35% (Table 3). 

**Table 3:** Serum biochemistry of participants S. SGOT: Serum glutamic-oxaloacetic transaminase, S. SGPT: Serum glutamic pyruvic transaminase, S. ALK. PHOS: Serum alkaline phosphatase

Investigations		Number	Percentage
Hypoglycemia	Absent	90	90.0
	Present	10	10.0
Serum Bilirubin	Normal	77	77.0
	Raised	23	23.0
Serum Albumin	Normal	79	79.0
	Low	21	21.0
Serum Urea	Normal	80	80.0
	Raised	20	20.0
Serum Creatinine	Normal	72	72.0
	Raised	28	28.0
S. SGOT	Normal	65	65.0
	Raised	35	35.0
S. SGPT	Normal	65	65.0
	Raised	35	35.0
S. ALK. PHOS.	Normal	74	74.0
	Raised	26	26.0
Serum Sodium	Normal	75	75.0
	Hyper	14	14.0
	Hypo	11	11.0
Serum Potassium	Normal	79	79.0
	Hyper	4	4.0
	Hypo	17	17.0
Serum Calcium	Normal	76	76.0
	Hyper	4	4.0
	Hypo	20	20.0

Of the 100 patients in this study, 77 % were discharged/discharged on patient request, 15 left the hospital against medical advice, and eight patients expired (Table 4).

**Table 4:** Treatment outcome of participants DOPR: Discharged on patient request, LAMA: Left against medical advice

Outcome	Number	Percentage
Discharged	53	53
DOPR	24	24
LAMA	15	15
Expired	8	8
Survived	92	92
Expired	8	8

Mortality was higher in the younger age group, although there was no statistically significant relation between age and mortality. Similarly, the association between gender and mortality was not statistically significant. Conversely, the relation of serum albumin, serum sodium, and serum potassium with the survival of SAM was found to be statistically significant, as depicted in Table 5.

**Table 5:** Association of clinical and biochemical factors with survival in SAM SAM: Severe acute malnutrition

Clinical and biochemical characteristics of participants		Outcome			P-value (by chi-square/Fischer exact)
		Survived N=53 (%)	Expired N=8 (%)	Total N (61)	
Age	six to 12	24 (85.7)	4 (14.3)	28	0.075
	13 to 24	11 (73.3)	4 (26.7)	15	
	25 to 59	18 (100)	0	18	
Gender	Male	25 (86.2)	4 (13.8)	29	0.885
	Female	28 (87.5)	4 (15.2)	32	
Weight-for-height	< 2SD	9 (100)	0	9	0.207
	< 3SD	44 (84.6)	8 (15.4)	52	
Serum Albumin	Normal	45 (91.8)	4 (8.2)	49	0.021
	Low	8 (66.7)	4 (33.3)	12	
Hypoglycemia	Absent	47 (85.5)	8 (14.5)	55	0.316
	Present	6 (100)	0	6	
Serum Sodium	Normal	43 (93.5)	3 (6,5)	46	0.017
	Hypernatremia	4 (57.1)	3 (42.9)	7	
	Hyponatremia	6 (75)	2 (25)	8	
Serum Potassium	Normal	44 (93.6)	3 (6.4)	47	0.010
	Hyperkalaemia	2 (50)	2 (50)	4	
	Hypokalaemia	7 (70)	3 (30)	10	
Serum Calcium	Normal	43 (89.6)	5 (10.4)	48	0.407
	Hypercalcemia	2 (66.7)	1 (33.1)	3	
	hypocalcemia	8 (80)	2 (20)	10	

## Discussion

Severe acute malnutrition is predominantly seen in the period of infancy and childhood i.e., from six months up to five years of age. Severe malnutrition is not only an important cause of mortality and morbidity but also leads to permanent impairment of physical and possibly mental growth in those who survive. In a study by Chiabi et al. on the clinical spectrum of SAM among children in Cameroon, the median age was nine months and a nearly equal gender-wise distribution was observed with 50.8% male and 49.2% female [8]. Further, a similar sex distribution has been observed in some other studies [9,10].

In our study, 30% of the participants were completely immunized, 64% were partially immunized, and 6% were not immunized at all. Tariq et al. found that 13% of cases were completely immunized, 62.3% were partially immunized, and 24.6% were not immunized [11]. This variation in immunization status may be due to the implementation of Mission Indradhanush and other immunization programs as well as the increase in institutional deliveries in the state.

In this study, 33 children had dehydration, 22 had some dehydration, and 11 had severe dehydration with dehydration being the most frequent complication and is similar to the finding in the study by Chiabi et al. with an incidence of 29.6%. Grenov et al. also reported dehydration associated with mortality [12]. Furthermore, 12 children were found to have bilateral nutritional edema with nearly half of the cases being below one year. Similarly, bilateral nutritional edema was noted in 16.5% of patients in a study conducted by Sharma et al. [13], whereas no child was reported to have nutritional edema in the study by Ganesh et al.

Hypoglycemia was found in 10% of patients in this study while Gangaraj et al. reported only 3.9% of such cases [14]. Out of 100 patients in our study group, 14% had hypernatremia, while 11% had hyponatremia. A nearly similar distribution of hyponatremia in 11% and hypernatremia in 8.2% was found in the study by Tariq et al. Hyponatremia was seen in 43.4% in the study by Dakshayani et al. [15]. In the study by Meshram et al., hyponatremic children with SAM presented with dysnatremia in the form of hyponatremia in 56% and hypernatremia in 1.4% [16]. Hyponatremia was seen in 14% and hypernatremia in 19% of the children with SAM in the study by Lakshmi et al. [17]. Differences in the incidence of hyponatremia and hypernatremia cannot be clearly explained, although they may have been influenced by the morbidity for which the patient was admitted, including diarrhea, vomiting, etc. Out of 100 patients in our study group, 4% of patients had hyperkalemia while 17% had hypokalemia. Mortality among those with normal potassium levels was less than 4%; however, when serum potassium levels were altered, mortality increased to about 50% in cases with hyperkalemia and 17% in cases with hypokalemia. Hypokalemia was observed at 7.1% in Dakshayani et al.'s study [15]. In a study by Alasad et al. on the role of potassium in childhood mortality secondary to SAM, hypokalemia was evident in 70.2% of the patients and mortality was 3.1% in normokalemic and 13.9% in hypokalemic patients [18]. However, hyperkalemia was not considered in both of these studies. Hypokalemia occurred in 44.3% of cases in the study by Okposio et al. [19]. Out of 100 patients, four had hypercalcemia while 20 had hypocalcemia. In a study on serum sodium, potassium, and calcium levels in children aged six to 59 months with SAM by Fatima et al., hypocalcemia and hypercalcemia were considered if serum calcium was less than 7.5 mg/dl and more than 10.5 mg/dl, respectively. They found isolated hypocalcemia in 1.4% of cases only [20]. Our study found that serum sodium disturbances (p-value=0.037) and serum potassium disturbances (p-value=0.001) are associated with poor outcomes among severely malnourished children. Our study concluded that renal derangements (serum urea p-value=0.196 and serum creatinine p-value=0.215) are common among SAM children but weren't found to be significant. In our study, deranged liver function tests too were associated with substantial poor outcomes in terms of mortality but statistically not found to be significant. 

A widespread introduction of proper anthropometric tools will enable early and accurate diagnosis of SAM, and early detection and management are key to decreasing mortality and long-term sequelae in cases of SAM and co-morbidities as treatment delays will be reduced, disease transmission will decrease, case fatality rates will decrease, adverse sequelae will be prevented, and patients’ outcomes will improve. Also, early detection and dietary modification can lead to decreased mortality and morbidity.

One limitation of the study is that it was unicentric with a small sample size. Therefore, a multicentric study with a larger sample size is necessary for improving the result and with a follow-up of at least six months to one year. Also, there was no follow-up of the patients in this study, and as such, we could not predict the residual burden and sequelae of SAM. Therefore, further studies must be done with a long-term follow-up plan at multicentric levels for more generalizable results.

## Conclusions

Severe acute malnutrition is both a medical and social disorder, and the risk of mortality increases with severity. Also, confirmed cases represent only the tip of the iceberg of the whole burden of malnutrition. Children with SAM observe a slowing down of organ systems and undergo physiological and metabolic changes in an orderly sequence to allow survival on limited calories. Deranged liver function tests, renal function tests, and serum electrolytes are common findings and can act as prognostic indicators for severely malnourished children. Furthermore, high-risk cases can be identified and aggressively treated based on priority. Electrolyte disturbance is an important offending agent in the proper recovery of SAM patients from infections, as infections themselves may result in electrolyte disturbance. In addition, serum electrolyte disturbances in SAM are some of the most important predictors of the severity of the disease, and although sodium and potassium are the major electrolytes, the role of minor electrolytes such as magnesium, zinc, and vitamins cannot be neglected.
